The article "p-Akt as a potential poor prognostic factor for gastric cancer: a systematic review and meta-analysis" was published in 2017. Journal: Oncotarget.

# p-Akt as a potential poor prognostic factor for gastric cancer: a systematic review and meta-analysis

**DOI:** 10.18632/oncotarget.17001

**Published:** 2017-04-10

**Authors:** Fang Cao, Cong Zhang, Wei Han, Xiao-Jiao Gao, Jun Ma, Yong-Wei Hu, Xing Gu, Hou-Zhong Ding, Li-Xia Zhu, Qin Liu

**Affiliations:** ^1^ Department of General Surgery, Kunshan First People's Hospital Affiliated to Jiangsu University, Kunshan, Jiangsu 215300, P.R. China; ^2^ Department of Pharmacy, Kunshan Hospital of TCM, Kunshan, Jiangsu 215300, P.R. China; ^3^ Department of Pathology, Kunshan First People's Hospital Affiliated to Jiangsu University, Kunshan, Jiangsu 215300, P.R. China; ^4^ Department of Urological Surgery, Kunshan Hospital of TCM, Kunshan, Jiangsu 215300, P.R. China; ^5^ Department of Gynaecology and Obstetrics, Kunshan First People's Hospital Affiliated to Jiangsu University, Kunshan, Jiangsu 215300, P.R. China

**Keywords:** p-Akt, gastric cancer, prognosis, survival, meta-analysis

## Abstract

To understand the relationship between p-Akt expression and the prognosis of patients with gastric cancer, we searched six databases, Pubmed, EMBASE, Cochrane Library, CNKI, Wanfang and CBM for relevant articles in order to conduct this metaanalysis. The pooled hazard ratios and corresponding 95%CI of overall survival were calculated to evaluate the prognostic value of p-Akt expression in patients with gastric cancer. With 2261 patients combined from 13 available studies, the pooled HR showed a poor prognosis in patients with gastric cancer in the univariate analysis (HR=1.88, 95%CI:1.45-2.43, P<0.00001), and the group “univariate analysis+estimate” (HR=1.41, 95%CI: 1.01-1.97, P=0.04), but not in multivariate analysis (HR=0.66, 95%CI: 0.29-1.52, P=0.33) and estimate (HR=1.13, 95%CI: 0.65-1.95, P=0.67). In conclusion, our results indicated that p-Akt was likely to be an indicator of poor prognosis in patients with gastric cancer.

## INTRODUCTION

Gastric cancer, as one of the most dangerous diseases, has claimed countless lives in our accelerated society [1]. Although numerous markers implicated in gastric cancer have been identified, the prognosis remains to be dismal mainly due to marked heterogeneity in histologic characteristics and biological features [2]. In addition, patients at the same condition, such as histological grade, lymph node status and TNM staging, may have dissimilar clinical outcomes [3]. As a result, it is urgent to develop new reliable prognostic markers for patients with gastric cancer.

Akt, or protein kinase B, one of key proteins in the Akt/PI3K/PTEN signaling pathway, is a Serine/Threonine protein kinase that, once activated by phosphorylation, plays an important role in the process of malignant transformation [4]. Phosphorylated Akt (p-Akt) was implicated in inducing signals to interfere with the cell apoptosis, and promoting abilities of proliferation and motility through a crucial mechanism, the activation of mTOR (mammalian target of rapamycin) [4, 5, 6]. Overexpressed p-Akt was considered as an indicator of poor prognosis in many malignancies. For example, a recent meta-analysis reported that high p-Akt expression was significantly associated with worse overall survival in patients with breast cancer (HR=1.52, 95%CI:1.29–1.78, P=0.001) [7]. This prognostic value were also showed in another two meta-analyses which summarized a same conclusion that elevated p-Akt expression was related to poor survival in patients with non-small cell lung cancer [8, 9].

In gastric cancer, many trials also showed a negative relationship between p-Akt expression and survival. However, some studies failed to detect a significant relationship, and some even obtained a positive one. In particular, several trials gained contradictory results through univariate and multivariate analyses. Furthermore, there were no systematic reviews with meta-analysis about the prognostic value of p-Akt in gastric cancer.

In light of the outstanding controversy of p-Akt, we launched a systematic review of available studies with meta-analysis to evaluate the prognostic value of p-Akt in patients with gastric cancer.

## RESULTS

### Search results

As shown in Figure 1, a total of 2727 articles were retrieved in the initial search. In addition, 31 records were yielded by manual searching. After removing 264 duplicated studies, we read the titles and abstracts of the 2494 studies left, and then, excluded 2356 citations, leaving 138 studies for further full-text review. After punctiliously reading, 125 studies were excluded: 121 studies, including reviews or letters, were excluded for no or insufficient survival data; and four studies [10–13] were removed because they only investigated Akt expression, but not p-Akt. Therefore, 13 eligible studies [14–26] with 2261 patients in total, were enrolled finally in this meta analysis.

**Figure 1:** Flow chart for the selection of records to include

### Study characteristics

The basic characteristics and results of the 13 eligible studies were summarized in Table 1 and Table 2. Briefly, 11 studies were conducted in Asian populations, while the remaining used Caucasian populations [16, 20]; study sample sizes ranged from 28 to 424; all of the cohorts were treated with surgery, except one treated only with chemotherapy [20], and the treatment of another two studies was a combined regimen of surgery plus chemotherapy [17, 21]; p-Akt expression was detected in the cytoplasm or nucleus of the tissues in all the studies, with rabbit or mouse antibodies, and polyclonal or monoclonal antibodies, but two studies [23, 24] didn't reported what kind of p-Akt they used; the cut-offs were identified by the extent or intensity, but the cut-off values of p-Akt varied in each study. Seven of them selected a moderate value, such as 50%, score 3/6 and the median level, and five chose “>10%” according to the extent of the staining. However, the left one, “Murakami 2007”, considered the staining >1% as a positive value. Among all of them, five reported that high level of p-Akt expression was related to poor survival; and six revealed no significant impact on survival. However, two reported p-Akt as an indicator of good prognosis. Ten of these thirteen cohorts reported the relationship between p-Akt expression and overall survival. Among them, four gave a HR directly from univariate analysis, and another six only presented Kaplan–Meier survival curves with or without multivariate HRs. So, we estimated HRs from these six K-M curves.

**Table 1:** Characteristics of included studies

First author	Year	Region	Sample	Measure method	Age (years)	N. of M/F	Primary antibody	Treatment	Follow-up
Bian	2015	China	Tissue	IHC	NR	NR	Rabbit Ab	Surgery	Median 49 months
									(2-80months)
Chang	2015	Korea	Tissue	IHC	Mean 58.1	285/139	Rabbit pAb	Surgery	Mean 82.3 months;
					Median 61				Median96.1months
									(1 –131 months)
Cinti	2008	Italy	Tissue	IHC	34-83years	16/34	mAb	Surgery	at least 5 years
Han	2011	China	Tissue	IHC	Median 53	85/23	Rabbit pAb	Surgery	About 5 years
								Chemotherapy	
Kobayashia	2006	Japan	Tissue	IHC	NR	NR	Rabbit pAb	Surgery	>40 months
Liang	2015	China	Tissue	IHC	NR	NR	mAb	Surgery	>5 years
Luber	2011	Europe	Tissue	IHC	Median 63	30/9	Mouse mAb	Chemotherapy	Median 379 days
Murakami	2007	Japan	Tissue	IHC	Mean 70.8	84/56	Mouse pAb	Surgery	at least 5 years
								Chemotherapy	
Murayama	2009	Japan	Tissue	IHC	Median 65	77/32	Rabbit pAb	Surgery	Median 1953 days
									(50– 3197 days)
Nam	2003	Korea	Tissue	IHC	Mean 54.8	210/101	NR	Surgery	Mean 54 months
									(1-72 months)
Sasaki	2014	Japan	Tissue	Immunoblot	NR	NR	NR	Surgery	>5 years
Sukawa	2012	Japan	Tissue	IHC	Median 71	157/74	pAb	Surgery	About 10 years
Xue	2012	China	Tissue	IHC	Median65.5	158/71	Mouse pAb	Surgery	>5 years

N. of P.: the number of patients; M/F: male/female; mAb: monoclonal antibody; pAb: polyclonal antibody; NR: not reported.

**Table 2:** Characteristics of included studies

First author	Year	N. of P.	Location	Scoring method	Cut-off of p-Akt high expression	Outcome	Obtainment	HR	95%CI
Bian	2015	396	C	EI	Score 3-6	OS	U	1.931	1.379-2.703
						OS	M	1.332	0.943-1.882
						RFS	U	1.537	1.074-2.199
						RFS	M	1.221	0.847-1.762
Chang	2015	424	C	EI	>50%or moderate to strong intensity	DSS	M	0.724	0.485-1.083
Cinti	2008	50	C	E	>10%	RFS	K-M	3.04	1.18-7.85
Han	2011	108	CN	EI	Score >6	DFS	K-M	1.67	0.86-3.24
Kobayashia	2006	88	C	E	>50%	OS	K-M	2.16	0.86-5.43
Liang	2015	107	C	EI	Score >1.5	OS	K-M	1.78	1.09-2.91
						DFS	K-M	1.76	1.02-3.04
Luber	2011	28	N	E	>10%	OS	U	1.1	0.2-4.8
						TTP	U	0.5	0.1-1.5
Murakami	2007	140	CN	E	>1%	OS	M	0.227	0.119–0.433
						OS	K-M	1.63	0.64-4.10
Murayama	2009	109	C	EI	>10% or strongly stained	OS	M	0.35	0.11-1.16
						OS	K-M	0.16	0.04-0.64
			N			OS	M	1.787	0.80-3.99
			CN			OS	K-M	1.36	0.34-5.48
Nam	2003	311	C	E	Moderate to strong	OS	K-M	0.46	0.23-0.92
Sasaki	2014	40	CN	E	Median of the protein level	OS	U	2.453	0.945-6.368
						OS	M	0.572	0.236-1.389
Sukawa	2012	231	CN	E	>10%	OS	U	1.75	1.12-2.80
Xue	2012	229	CN	E	>10%	OS	K-M	1.73	1.16-2.59

N. of P.: the number of patients; C: cytoplasm; N: nucleus; CN: cytoplasm and nucleus; OS: overall survival; DFS: disease-free survival; DSS: disease-specific survival; TTP: time to progression; RFS: recurrence-free survival; HR: hazard ratio; “M”: the multivariate analysis; “U”: the univariate analysis; “K-M”: Kaplan–Meier survival curves; “E”: identifying the cut-off by the extent; “I”: identifying the cut-off by the intensity; “EI”: both by the extent and the intensity.

### Quality assessment

The study quality scores based on the NOS, ranged from 6 to 8, with a mean of 6.85. None of these thirteen studies obtained a NOS≤5, indicating that all of them had high levels of methodological quality in our meta-analysis (Table 3).

**Table 3:** Quality assessment of eligible studies with Newcastle-Ottawa Scale

First author	Year	NOS	Selection	Comparability	Outcome
Bian	2015	6	★★★*	★	★★*
Chang	2015	8	★★★	★★	★★★
Cinti	2008	7	★★★	★★	★★
Han	2011	7	★★★*	★*	★★★
Kobayashia	2006	6	★★★	★	★★*
Liang	2015	6	★★*	★★*	★★*
Luber	2011	7	★★★	★	★★★*
Murakami	2007	8	★★★	★★	★★★*
Murayama	2009	8	★★★	★★*	★★★
Nam	2003	6	★★★*	★★	★*
Sasaki	2014	7	★★	★★	★★★*
Sukawa	2012	7	★★★*	★	★★★*
Xue	2012	6	★★★	★*	★★

*The score was produced by discussion.

### p-Akt expression and survival outcome

16 results, obtained from ten trials with OS, were divided into three groups, univariate, multivariate and estimate, by which three pooling HRs were produced (HR=1.88, 95%CI:1.45-2.43, P<0.00001; HR=0.66, 95%CI: 0.29-1.52, P=0.33; and HR=1.13, 95%CI: 0.65-1.95, P=0.67, respectively. Figure 2). However, only the group, univariate, with a I^2^=0%, had no heterogeneity. Then, we combined the two groups, univariate and estimate, and figured out a new incorporative HR being 1.41 (95%CI: 1.01-1.97, P=0.04, Figure 2D). Though with highly significant heterogeneity (I^2^=62%, Ph=0.004), this new result also had significance in statistics, illustrating that high p-Akt expression was significantly associated with poor OS of patients with gastric cancer.

**Figure 2:** Forest plot of hazard ratios (HRs) for OS of high p-Akt expression versus low expression in gastric cancer **(A)** The HRs for OS in univariate analysis; **(B)** the HRs for OS in multivariate analysis; **(C)** the HRs for OS in estimate; **(D)** the HRs for OS in univariate analysis and estimate.

We also calculated the pooled HRs of DFS and RFS, and obtained statistically significant estimates (HR=1.72, 95%CI: 1.13-2.63, P=0.01; and HR=1.67, 95%CI: 1.20-2.34, P=0.003, respectively), showing elevated p-Akt expression associated with poor prognosis. However, we failed to obtain more pooling HRs of other survival outcomes.

### Subgroup analyses

Due to the heterogeneity, we performed the subgroup analyses, presented in Table 4, by stratifying the combined data according to location (C vs. N vs. CN), main treatment (surgical vs. non-surgical), study region (Asian vs. Caucasian), sample size (<100 vs. ≧100), obtainment (univariate vs. estimate), scoring method (E vs. EI), cut-off (1% vs. 10% vs. Moderate), measure method (IHC vs. Immunoblot) and primary antibody (Rabbit vs. Mouse vs. pAb vs. mAb vs. NR). Because of too few cohorts in multivariate analysis, and no heterogeneity in univariate analysis, we conducted the subgroup analyses only in the combination of univariate analysis and estimate, called “U+E”, and we failed to get any potential source of heterogeneity in “U+E”.

**Table 4:** Subgroup analyses of the association between high p-Akt expression and overall survival in the group “U+E” of patients with gastric cancer

Subgroup	Data sets	Model	HR (95%CI)	P	I^2^	Ph
All	11	Random	1.41 [1.01, 1.97]	0.04	62%	0.004
Location						
C	5	Random	1.04 [0.51, 2.10]	0.92	84%	<0.0001
N	1	-	1.10 [0.20, 6.05]	0.91	-	-
CN	5	Fixed	1.76 [1.35, 2.30]	<0.0001	0%	0.96
Region						
Asian	10	Random	1.42 [1.00, 2.01]	0.05	65%	0.002
Caucasian	1	-	1.10 [0.20, 6.05]	0.91	-	-
Treatment						
Surgical	10	Random	1.42 [1.00, 2.01]	0.05	65%	0.002
Non-surgical	1	-	1.10 [0.20, 6.05]	0.91	-	-
Sample size						
<100	3	Fixed	2.09 [1.12, 3.87]	0.02	0%	0.72
≧100	8	Random	1.28 [0.86, 1.91]	0.22	72%	0.0009
Obtainment						
univariate	4	Fixed	1.88 [1.45, 2.43]	<0.00001	0%	0.85
estimate	7	Random	1.13 [0.65, 1.95]	0.67	73%	0.001
Scoring method						
E	7	Random	1.46 [0.96, 2.21]	0.08	57%	0.03
EI	4	Random	1.21 [0.60, 2.44]	0.59	75%	0.008
Cut-off						
1%	1	-	1.63 [0.64, 4.15]	0.31	-	-
10%	5	Random	1.19 [0.65, 2.18]	0.57	64%	0.03
Moderate	5	Random	1.51 [0.89, 2.56]	0.13	73%	0.005
Measure method						
IHC	10	Random	1.35 [0.95, 1.92]	0.10	64%	0.003
Immunoblot	1	-	2.45 [0.94, 6.37]	0.07	-	-
Primary antibody						
Rabbit	4	Random	1.13 [0.45, 2.85]	0.79	75%	0.007
Mouse	3	Fixed	1.68 [1.17, 2.41]	0.005	0	0.88
pAb	1	-	1.75 [1.12, 2.73]	0.02	-	-
mAb	1	-	1.78 [1.09, 2.91]	0.02	-	-
NR	2	Random	1.03 [0.20, 5.29]	0.97	87%	0.005

C: cytoplasm; N: nucleus; CN: cytoplasm and nucleus; U+E: univariate analysis + estimate of Kaplan–Meier survival curves.

### p-Akt expression and clinicopathological features

In our study, we also assessed the relationship of p-Akt expression with pathological differentiation, N status and tumor staging. In spite of no significant difference between p-Akt expression and pathological differentiation, we found that high p-Akt expression was associated with lymph node metastasis and advanced gastric cancer (for pathological differentiation, HR=1.17, 95%CI: 0.94-1.46, P=0.15; for N status, HR=1.34, 95%CI: 1.11-1.62, P=0.003; and for tumor staging, HR=1.60, 95%CI: 1.27-2.02, P<0.0001).

### Sensitivity analyses

By using sensitivity analysis, we deleted an individual result at a time and pooled the others into a new HR to compare with the previous one, and all studies of this meta-analysis were assessed to value the stability of our results. Pooled results for “univariate”, “multivariate” and “estimate” were insensitive to the removal of individual studies, and the corresponding combined HRs were not substantially changed (data not shown, Figure 3).

**Figure 3:** Influence analysis **(A)** was about univariate analysis; **(B)** was about multivariate analysis; **(C)** was about estimate.

### Publication bias

We conducted the publication bias assessment of the thirteen studies by funnel plots and Egger's test. No obvious asymmetry was found in all of the three groups (Figure 4), and results of Egger's test also suggested no evidence of publication bias in “univariate”, “multivariate” and “estimate” (P=0.752, P=0.367 and P=0.278, respectively).

**Figure 4:** Funnel plot of 10 studies **(A)** was about univariate analysis; **(B)** was about multivariate analysis; **(C)** was about estimate.

## DISCUSSION

p-Akt, as a potential biomarker of poor prognosis in various malignant tumors, has aroused prominent interest in this critical period of high morbidity and mortality of neoplasms. Although some studies failed to find any significance of the relationship between p-Akt expression and survival, all of these three meta-analyses proved that over-expression of p-Akt was correlated with an unfavorable outcome in carcinomas [7, 8, 9]. In spite of small sample sizes and controversial reports, many studies have investigated the prognostic value of p-Akt in gastric cancer. Furthermore, no meta-analyses have previously been conducted on the prognostic value of p-Akt in gastric cancer. Hence, we performed this meta-analysis to clarify this question and explore its prognostic value in gastric cancer.

To the best of our knowledge, the present meta-analysis, including a total of 13 studies with 2261 patients, was the first meta-analysis systematically evaluating the prognostic value of p-Akt in patients with gastric cancer, and showed that over-expressed p-Akt was a strong predictor of inferior overall survival in the univariate analysis in patients with gastric cancer. Though without any significance in multivariate analysis and estimated K-M curves, a poor prognosis associated with high p-Akt expression could be found in the group, “U+E”, which we pooled results obtained from studies in the group of univariate analysis, and those in the group of estimate. Because those estimates calculated form curves was univariate, but not multivariate, we also figured out estimates from K-M curves of studies only with multivariate analysis [8]. In our following sensitivity analysis, no substantial changes were found, and another strength of this meta-analysis was that no publication biases were detected, indicating that our combined results may be unbiased. In our study, we also found that high p-Akt expression was correlated with lymph node metastasis and advanced gastric cancer.

Many molecular mechanisms, associated with the alteration of p-Akt expression in malignancies, have been explored out. In a total of 202 gastric cancer patients, Hisamatsu demonstrated that there was a positive relationship between p-Akt and EGFR, both of which were significantly correlated with DNA aneuploidy [27]. The signaling pathway, Akt/PI3K/PTEN/mTOR, was related to the pathogenic process of several neoplastic diseases [28, 29], and the activation of this signaling pathway was also associated with poor survival in solid tumors [30]. Many molecular biomarkers, such as SPARC, ZIC1 and NM23-H1, were up-regulated or down-regulated through the Akt/PI3K/PTEN/mTOR signaling pathway, and promoted or inhibited the growth of human tumors [31–33]. Besides, overexpression of these proteins might also be linked to better or worse survival [34–36]. Moreover, some drugs, such as 5-FU and LY294002, could downregulate the activated p-Akt to overcome intrinsic and acquired resistance of 5-FU in SNU-719 cells, a EBV gastric cancer cell line [37]. Therefore, this pro-oncogenic signal, p-Akt, the prognostic value of which will be more important, especially with respect to Akt/PI3K/PTEN/mTOR signaling pathway, has become a promising target for the development of drugs.

Admittedly, several limitations were unavoidable in our meta-analysis. Firstly, though with 2261 patients in total, the sample size was still small. The studied patients couldn't reflect the real outcome of whole gastric cancer population and this could cause some selection bias or else. Secondly, despite the HRs estimated from Kaplan-Meier curves were results of univariate analysis, these estimates were inaccurate and might influence our results in the groups, estimate and “U+E”. In addition, although many meta-analyses combined HRs whether with univariate analysis or with multivariate analysis, our study considered that HRs with univariate analysis, including estimated from univariate curves, included some confounding factors, but HRs with multivariate analysis precluded these factors, to some degree. Although HRs with multivariate analysis seemed to be better, the capability to eliminate factors of each study must be different. Thus, all groups should be calculated and discussed in our manuscript. Thirdly, Meta-analysis is an effective method to combine the results of RCT, but recently, this approach has been applied successfully for evaluation of prognostic indicators in patients with malignant diseases. However, these studies investigating genes expression couldn't be designed as RCT, so all studies were non-RCT. Fourthly, although we obtained a significant pooled HR without any heterogeneity when deleting two studies, “Nam 2003” and “Murayama 2009 C”, in the sensitivity analysis, we failed to find the potential source of heterogeneity in the subgroup analyses, which meant that various factors might be lumped together. So, some possible sources of heterogeneity might be undetected. Fifthly, in our subgroup analyses, Akt expression seemed to correlate with prognostic outcome only in studies conducted in Asian countries or surgical treatment (only one study conducted in Caucasian and non-surgical treatment). Besides, the cut-offs were various and we divided them into three parts, “>1%”, “>10%” and “moderate”, but we failed to gain any significant HR, and the heterogeneity was still existent. Thus, the pooling HR combined by results with univariate analysis and results estimated by K-M curves might be unstable, and more researches, with a standard cut-off, on p-Akt expression in gastric cancer should be conducted. In addition, some unpublished studies and negative studies could also be ignored. Because we launch this rigorous search to collect as many studies as possible, and then funnel plots and Egger's test both showed no obvious publication bias in our results, the influence of these studies might be limited. Last but not least, we only searched the studies in English and Chinese. This could lose some available studies in other languages.

In conclusion, the elevated p-Akt expression might be associated with a poor prognosis in patients with gastric cancer. This meta-analysis showed the current status of many inconsistencies and imperfections in researches of p-Akt in gastric cancer. Thus, more rigorous studies should be performed to confirm our conclusion and explore its molecular functions.

## MATERIALS AND METHODS

### Publication selection

We searched Pubmed, EMBASE, Cochrane Library, CNKI (China National Knowledge Infrastructure), Wanfang (Chinese database) and CBM (China Biological Medicine Database) from their incipiency to January, 2016. The key words were used as follow: “Akt”, “phospho-Akt”, “protein kinase B”, “PKB”, “gastric”, “stomach”, “prognosis” and “survival”. Reference lists of reviews and articles were hand-searched for potential articles. Also, manuscripts were manually scrutinized to obtain additional trials most relevant to this review. Only studies published in peer reviewed journals in English or Chinese were included. All the initially identified articles were scanned independently by two reviewers (Fang Cao and Cong Zhang). However, we had no protocol developed for this review.

### Inclusion and exclusion criteria

Inclusion criteria were: (a) clinical trials reported patients with gastric cancer; (b) p-Akt protein expression in the tissue specimens of patients with gastric cancer, was measured with immunohistochemistry (IHC) or immunoblot analysis; (c) studies reported the association between p-Akt expression and survival outcome; (d) studies contained HRs and 95% CI for OS or other outcomes which either were reported or could be estimated from K-M curves; (e) if the study population was overlapping or duplicated, only the most recent or the most complete report would be enrolled.

Exclusion criteria were: (a) experiment only *in vitro* or *in vivo* but not based on patients; (b) literature published as abstracts, letters, reviews, editorials, case reports and expert opinions; (c) studies without HRs and its corresponding 95%CI about OS, or K-M survival curves; (d) studies only with data about mutations of the Akt gene or only reporting mRNA; (e) similar and repeated studies.

Disagreement was resolved by discussion between two reviewers (Fang Cao and Cong Zhang) or consultation with a third one (Wei Han).

### Data extraction and quality assessment

We extract the following information from each study: (a) general information, including first author, publication year, region of origin, sample size, gender and age of patients, and the follow-up duration; (b) clinical outcomes, including OS or others, with HRs and 95%CI. If no univariate or unadjusted HR was available, we used a digitizing program, Engauge Digitizer, which could rendered K-M curves into numbers. And then, we put the data into a Tierney table, by which the estimated HR with its corresponding 95%CI were figured out immediately [38]. This estimate was performed independently by two reviewers (Fang Cao and Cong Zhang), and the disagreement was also resolved by discussion between the two reviewers or consultation with a third reviewer (Wei Han). Note that, despite we obtained univariate unadjusted HRs, multivariate adjusted HRs and estimated HRs, we only combined univariate unadjusted HRs and estimated HRs into a new pooled estimate, rather than the multivariate adjusted HRs [8].

Two independent reviewers (Fang Cao and Cong Zhang) assessed the quality of each study with the Newcastle-Ottawa Quality Assessment Scale (NOS) [39]. This scale, including three parts, selection, comparability and outcome, mainly used in non-RCT studies. We used the quality assessment scale of cohort studies. A study with NOS ≥ 6 was regarded as a high-quality study [40]. Disparity was also resolved by discussion or consultation.

### Data synthesis and analysis

OS (overall survival), associated with p-Akt expression in patients with gastric cancer, was the primary outcome. Other survival outcomes, including DFS (disease-free survival), TSS (tumor-special survival), DSS (disease-specific survival), TTP (time to progression), MFS (metastasis-free survival) and RFS (recurrence-free survival), were also collected. HR with its 95% CI was used to be the effect measure of interest. Estimates of HRs were weighted and pooled using the Mantel-Haenszel method. A pooled HR>1.00, with its 95%CI did not overlap 1, indicated a worse survival for the group with p-Akt expression.

The Q and I^2^ test were used to measure the heterogeneity among cohorts. A random or Fixed model was identified by the heterogeneity analysis. A fixed effect model was selected if I^2^<50%; and the random effect model was applied if I^2^≧50%. An I^2^>50% indicated substantial heterogeneity in studies, and we would perform subgroup analyses to detect potential sources of heterogeneity.

A funnel plot and Egger's linear regression test were used to assess the latent publication bias, and in Egger's test, a value <0.05 indicated an inevitable significant publication bias [41].

All the analyses were conducted by STATA statistical software package version 12.0 (STATA12) and Review Manager software version 5.3 (The Cochrane Collaboration, RevMan5.3). All statistical tests were two-tailed and P<0.05 was considered statistically significant.
